The article "Bioinformatic Analysis of Immune Significance of RYR2 Mutation in Breast Cancer" was published in 2021. Journal: Biomed Res Int.

# Bioinformatic Analysis of Immune Significance of RYR2 Mutation in Breast Cancer

**DOI:** 10.1155/2021/8072796

**Published:** 2021-11-03

**Authors:** Zhiquan Xu, Ling Xiang, Rong Wang, Yongfu Xiong, He Zhou, Haitao Gu, Jijian Wang, Linglong Peng

**Affiliations:** ^1^Department of Gastrointestinal Surgery, The Second Affiliated Hospital of Chongqing Medical University, Chongqing 400010, China; ^2^Department of Clinical Nutrition, The Second Affiliated Hospital of Chongqing Medical University, Chongqing 400010, China; ^3^Department of Oncology, The Fifth Affiliated Hospital of Sun Yat-sen University, Zhuhai 519000, China; ^4^Department of Hepatobiliary Surgery, The Affiliated Hospital of North Sichuan Medical College, Sichuan 637000, China; ^5^Department of Gastrointestinal Surgery, The Affiliated Hospital of North Sichuan Medical College, Sichuan 637000, China

## Abstract

**Background:**

Currently, immunotherapy is widely used for breast cancer (BC) patients, and tumor mutation burden (TMB) is regarded as a valuable independent predictor of response to immunotherapy. However, specific gene mutations and their relationship with TMB and tumor-infiltrating immune cells in BC are not fully understood.

**Methods:**

Comprehensive bioinformatic analyses were performed using data from The Cancer Genome Atlas (TCGA) and International Cancer Genome Consortium (ICGC) datasets. Survival curves were analyzed via Kaplan-Meier analysis. Univariate and multivariate Cox regression analyses were used for prognosis analysis. Gene set enrichment analysis (GSEA) was performed to explore regulatory mechanisms and functions. The CIBERSORT algorithm was used to calculate the tumor-infiltrating immune cell fractions.

**Results:**

We analyzed somatic mutation data of BC from TCGA and ICGC datasets and found that 19 frequently mutated genes were reported in both cohorts, namely, SPTA1, TTN, MUC17, MAP3K1, CDH1, FAT3, SYNE1, FLG, HMCN1, RYR2 (ryanodine receptor 2), GATA3, MUC4, PIK3CA, KMT2C, TP53, PTEN, ZFHX4, MUC16, and USH2A. Among them, we observed that RYR2 mutation was significantly associated with higher TMB and better clinical prognosis. Moreover, GSEA revealed that RYR2 mutation-enriched signaling pathways were related to immune-associated pathways. Furthermore, based on the CIBERSORT algorithm, we found that RYR2 mutation enhanced the antitumor immune response by enriching CD8+ T cells, activated memory CD4+ T cells, and M1 macrophages.

**Conclusion:**

RYR2 is frequently mutated in BC, and its mutation is related to increased TMB and promotes antitumor immunity; thus, RYR2 may serve as a valuable biomarker to predict the immune response.

## 1. Introduction

Breast cancer (BC) is the most common malignancy in women worldwide, with approximately 2.1 million new cases in 2018 [1]. Although current comprehensive treatments for BC, including surgery, chemotherapy, radiotherapy, endocrine therapy, and targeted drug therapy, have significantly improved the survival rate of patients, some patients still develop tumor recurrence due to drug resistance and eventually die [2]. In recent years, the discovery of immune checkpoints has opened a new era in the treatment of malignant tumors [3]. In clinical practice, immune checkpoint inhibition targeting programmed cell death receptor 1 (PD-1) and its ligand PD-L1 has been applied to a variety of solid tumors and significantly improved the overall survival (OS) of patients [4]. Currently, the American Food and Drug Administration (FDA) has approved atezolizumab (an inhibitor of PD-L1) in combination with albumin paclitaxel for first-line treatment of advanced triple-negative breast cancer (TNBC). However, BC is a “cold” tumor in immunotherapy [5]. In terms of overall efficacy, BC patients do not benefit as much from immunotherapy as patients with other solid tumors, such as non-small-cell lung cancer and melanoma [6]. Thus, the use of effective immune markers to screen out BC patients who are more likely to benefit from immunotherapy is an important research direction. The most critical problem for BC immunotherapy is how to choose the appropriate population and reasonable predictors of immunotherapy efficacy to prolong the survival time of patients and improve their quality of life.

The PD-1/PD-L1 signaling pathway is the most intensively studied pathway in immunotherapy [7]. Tumor cells achieve immune escape using the PD-1/PD-L1 signaling pathway to evade immune monitoring. Both tumor cells and immune cells can overexpress PD-L1. When PD-1 on the surface of T cells binds to PD-L1, the immune response of T cells to tumor cells is inhibited, enabling tumor cells to escape being killed by the immune system [8, 9]. PD-1 or PD-L1 antibodies can block the binding between PD-1 and PD-L1 and reactivate the immune response of T cells to tumor cells [8]. Thus, high PD-L1 expression is considered a good indicator for tumor immunotherapy. A meta-analysis of advanced BC showed that PD-L1 not only is related to the prognosis of advanced BC patients but also is a biomarker for screening the appropriate population for immunotherapy [10]. Although the expression level of PD-L1 in tumors can be clinically assessed by immunohistochemistry, PD-L1 expression in tumors is heterogeneous and affected by previous chemotherapy and radiotherapy [11, 12]. In addition, the methods for PD-L1 detection and the critical value of positive PD-L1 expression are not standardized [13]. Thus, the use of PD-L1 as a biomarker for immunotherapy sensitivity is still limited.

Tumor mutation burden (TMB) is the total number of nonsynonymous somatic cell mutations in tumor cells [14]. Nonsynonymous mutations can produce neoantigens recognized by the host immune system, thus triggering removal by the immune system and inducing the host immune response to scavenge tumor cells [15]. Therefore, tumor cells with higher levels of TMB may be more easily recognized by the immune system, which in turn triggers a stronger immune response to checkpoint inhibitors [16]. It has been confirmed that high TMB is associated with high tumor immunogenicity in different types of tumors, and the clinical response and survival rate of high TMB tumors, such as melanoma, lung cancer, and colorectal cancer, are significantly increased [17]. In a clinical trial, TMB was more significantly correlated with response rates than the expression level of PD-L1 [18]. These results suggest that TMB can be used as a tumor predictor of clinical benefit and a prognostic factor and that it has the potential to play a key role in predicting the efficacy of immune checkpoint inhibitors. A recent study analyzed clinical research data on PD-1 inhibitors and PD-L1 inhibitors in 27 solid tumor types, including BC, and found that TMB was significantly positively correlated with the objective response rate to immunotherapy [19]. TMB expression was significantly different among different gene mutation subtypes of BC. TMB expression was highest in TNBC patients, followed by HER2-positive patients, while TMB expression was lowest in patients with estrogen receptor- (ER-) positive, progesterone receptor- (PR-) positive, and human epidermal growth factor receptor-2- (HER2-) negative BC subtypes [20]. At present, whether TMB can directly predict the efficacy of immunotherapy for BC is still controversial, but some studies suggest that patients with a high TMB have a better prognosis when stratified by gene mutation and analyzed in combination with immune subtypes [21]. Therefore, high TMB-related gene mutation analysis may be a good predictor of immunotherapy efficacy, which can contribute to screening for the appropriate population for BC immunotherapy. However, specific gene mutations and their relationship with TMB and tumor-infiltrating immune cells in BC are not clear. Thus, this study is aimed at exploring whether TMB and prognosis-related genes are closely related to BC immunotherapy.

## 2. Materials and Methods

### 2.1. Data Acquisition

A total of 1222 RNA expression profile samples of BC were downloaded from TCGA database (http://portal.gdc.cancer.gov/projects), including 1109 tumor samples and 113 normal samples. The clinical information of 1097 patients with BC was downloaded from TCGA database. After excluding those patients with missing clinical data, 980 samples were used for further analysis. The somatic mutation data of 877 United States patients from TCGA database and 508 European Union patients from the ICGC database (http://dcc.icgc.org/releases/current/Projects) were downloaded and extracted in Perl software so that it can be analyzed in R software.

### 2.2. Classification of BC Based on TMB

TMB was defined as the total number of somatic gene coding errors, gene insertions, gene deletions, and base substitutions detected per million bases. As described in previously published research, only mutations that cause changes in amino acids were counted [14].

### 2.3. Bioinformatic Analysis

As described in a previous study [22], R (v4.0.2) was used for bioinformatic analysis. The 30 genes with the highest mutation frequency in TGCA and IGGC databases were extracted with Perl. Somatic mutation data for both American and European Union BC samples were processed and visualized with the “GenVisR” package [23]. The R package “venn” was used to screen for the same mutated genes in both databases. The association between mutated genes and TMB was analyzed and visualized using the R package “ggpubr.” Due to the lack of survival information in the ICGC database, patients from TCGA database were sorted into two groups according to gene mutation states. Survival curves were analyzed and visualized using the R packages “survminer” and “survival.” Gene set enrichment analysis (GSEA) was performed with GSEA software (v4.1.0), and the conditions set included normalized enrichment score (NES) = 1000 and FDR *p* value < 0.05 [24]. The selected gene sets for GSEA contained “c5.go.bp.v7.2.symbols.gmt,” “c5.go.cc.v7.2.symbols.gmt,” and “c5.go.mf.v7.2.symbols.gmt.” The CIBERSORT algorithm was used to estimate the relative abundance of immune cell infiltration in patients with different *RYR2* statuses [25]. The number of permutations was set to 1000, and a threshold *p* value of <0.05 was the criterion for the successful computation of a sample. Matrix data visualization was performed with the R package “corrplot.” Difference analysis of infiltrating immune cells between the *RYR2-*mutant and *RYR2-*wild-type groups was performed using the R package “limma” and visualized with the R package “vioplot.”

### 2.4. Statistical Analysis

Statistical analyses were performed with R software (version 4.0.2). Survival curves were analyzed using Kaplan-Meier survival analysis and a log-rank test. Univariate and multivariate Cox regression analyses were used for prognosis analysis. The correlation between mutant genes and TMB was analyzed with a Mann–Whitney *U* test. For all comparisons, a two-tailed *p* value < 0.05 was considered statistically significant.

## 3. Results

### 3.1. Landscape of Somatic Mutations in BC

We first analyzed the mutations of the top 30 genes with high mutation frequency in TCGA database (*n* = 877). As shown in Figure 1(a), the mutation spectrum of the top 30 genes was mainly missense mutations, and the five genes with the highest mutation frequencies were *PIK3CA* (36.7%), *TP53* (35.8%), *TTN* (17.8%), *CDH1* (13.0%), and *GATA3* (11.3%). We then analyzed the genetic mutation profiles of BC patients in the European Union in the ICGC database (*n* = 508). The top 30 frequently mutated genes with high mutation frequency and the pattern of somatic mutation for the top 30 genes are illustrated in Figure 1(b), among which the five most frequently mutated genes were *TP53* (35.6%), *PIK3CA* (29.9%), *TTN* (18.9%), *GATA3* (8.1%), and *MAP3K1* (7.5%).

### 3.2. Gene Mutations Associated with TMB

We further screened out genes with high mutation frequency in both databases via a Venn diagram. Our results demonstrated that 19 frequently mutated genes reported in TCGA cohort were also reported in the ICGC cohort, namely, *SPTA1*, *TTN*, *MUC17*, *MAP3K1*, *CDH1*, *FAT3*, *SYNE1*, *FLG*, *HMCN1*, *RYR2*, *GATA3*, *MUC4*, *PIK3CA*, *KMT2C*, *TP53*, *PTEN*, *ZFHX4*, *MUC16*, and *USH2A* (Figure 2(a)). To further investigate the relationship between these highly mutated genes and TMB, the TMB value of each patient in TCGA database was calculated, and patients were assigned to the wild-type group or mutation group based on the 19 gene mutation statuses. The TMB score in BC ranged from 0.03 to 118.45 per Mb, with a median of 1.56 per Mb. As shown in Figure 2(b), among these high-frequency mutated genes in both databases, 14 of the 19 genes, including *RYR2*, with a mutation type had a higher TMB value than those genes with the wild type. Interestingly, patients with mutations in *MAP3K1* showed a lower TMB, and there was no significant difference in TMB between the mutation group and the wild-type group of the other 4 genes (*CDH1*, *GATA3*, *PIK3CA*, and *KMT2C*) (Figure 2(b)).

### 3.3. *RYR2* Mutation Associated with Prognosis

A previous study reported that higher TMB indicated favorable overall survival in BC patients [26]. To identify prognosis-related gene mutations, Kaplan-Meier analysis was performed on the TMB-related commonly mutated genes. The results demonstrated that only *RYR2* mutation (HR = 0.140; 95% CI, 0.020–1.000; *p* = 0.021) was associated with a better prognosis (Figure 3). However, the *RYR2* mutation did not remain statistically significant after considering age, sex, TNM classification, and TMB status in the Cox regression model (Figure 4).

### 3.4. Identification of Enrichment Pathways for Patients with *RYR2* Mutation

It is well known that TMB is an important indicator to judge the efficacy of tumor immunotherapy [17]. Thus, we next investigated whether *RYR2* mutation-enriched signaling pathways are related to immunity. GSEA was performed, and the results showed that pathways were significantly enriched in the *RYR2* mutant group, including antigen processing and presentation; antigen processing and presentation of peptide antigen via MHC class I/II, MHC class I/II protein binding, and NF-*κ*B binding; regulation of response to IFN-*γ*; and response to IL-12. These results suggest that certain immune-related pathways are associated with *RYR2* mutations in BC patients (Figure 5).

### 3.5. Tumor-Infiltrating Immune Cells Associated with *RYR2* Mutation in BC

According to the CIBERSORT algorithm, we further assessed the association between *RYR2* mutation and tumor-infiltrating immune cells in the BC microenvironment. Our results demonstrated that the composition of 22 immune cell types in each sample varied significantly, and the infiltrating immune cells were mainly T cells and macrophages in BC samples (Figure 6). In addition, we observed that CD8 T cells, native CD4 T cells (low infiltration in both the *RYR2* mutant and wild-type groups), activated memory CD4 T cells, and M1 macrophages were more enriched in the *RYR2* mutant-type group than in the wild-type group (Figure 7(a)). Furthermore, the correlation matrix results revealed that CD8 T cells had the strongest positive correlation with activated memory CD4 T cells and M1 macrophages but were negatively correlated with M2 macrophages (Figure 7(b)). Moreover, M1 macrophages were positively associated with activated memory CD4 T cells and CD8 T cells and negatively correlated with M2 macrophages (Figure 7(b)).

## 4. Discussion

In our study, our data suggest that TMB and the prognosis-related gene RYR2 are closely related to the immune response of BC. These results support previous findings that these immune cells play a major role in the tumor microenvironment and enhance the immune response against tumor immune escape [27–29].

Intracellular calcium ions (Ca^2+^) play an important role in basic cellular physiology [30]. Accumulating evidence has shown that intracellular Ca^2+^ homeostasis is disrupted in tumor cells, and these changes are involved in genetic mutations, cancer cell proliferation, apoptosis, and migration [31–33]. *RYR2* is a member of the *RYR* family and a major component of the Ca^2+^ pathway, which regulates the release of Ca^2+^ from the sarcoplasmic reticulum into the cytoplasm [34]. In an *RYR2*-positive prostate cancer cell line, *RYR*-related Ca^2+^ mobilization augments tumor cell apoptosis [35]. Moreover, *RYR2* expression is correlated with poor prognosis in patients with thyroid carcinoma [36], and strong *RYR2* upregulation was found in a BC cell line upon EGF-induced epithelial-to-mesenchymal transition [37]. In addition to *RYR2* expression alteration, a high *RYR2* mutation frequency is a common feature of numerous human malignancies. *RYR2* somatic mutation is widely observed in cervical cancer patients, and it is speculated that *RYR2* can be used as a target for cervical cancer treatment [38]. Cai et al. reported that *RYR2* is a frequently mutated gene with predicted neoantigens presented by MHC class I and class II molecules and thus is a candidate for lung adenocarcinoma immunotherapy [39]. Schmitt et al. demonstrated that impaired *RYR2* function due to somatic mutation is a common event in the pathogenesis of head and neck cancer [40]. For BC, *RYR2* mutation was found to be correlated with a decreased BC risk restricted by PR, ER, and tumor stage [41]. In the present study, we found that *RYR2* mutation was associated with a favorable prognosis and increased TMB in BC patients. TMB is the total number of somatic gene coding errors, gene insertions, gene deletions, and base substitutions detected per million bases [14]. High TMB in tumor cells produces more neoantigens that can be recognized by the host immune system and trigger the immune response [19, 42]. Thus, we speculate that *RYR2* mutation with a high TMB in BC might drive the immune system to scavenge tumor cells.

The tumor microenvironment plays an important role in the occurrence and development of BC [43]. The immune microenvironment, composed of tumor-infiltrating lymphocytes, tumor-related macrophages, and other immune cells, is an important part of the tumor microenvironment [44]. Under the influence of different cellular activation mechanisms and cytokines, tumor-infiltrating immune cells produce different immune responses, which can directly reflect the local immune response of the tumor microenvironment [45]. The tumor-infiltrating immune cells in BC mainly derive from the tertiary lymphoid structure and are dominated by two opposing forces [46]. One is antitumor cells mainly composed of CD4+ Th1 cells, CD8+ cytotoxic T lymphocytes (CTLs), NK cells, M1 macrophages, and dendritic cells, while the other is capable of promoting tumor growth and includes CD4+ FOXP3+ T cells (Tregs), CD4+ Th2 cells, and M2 macrophages [47]. In our study, we found that samples with *RYR2* mutation were more infiltrated by CD8 T cells, activated memory CD4 T cells, and M1 macrophages than samples with wild-type *RYR2*, indicating that *RYR2* mutation may promote antitumor immunity in BC patients. This finding is in line with previous evidence indicating that *RYR2* mutation and its transcriptomic signature are associated with a favorable outcome and immune infiltrates in basal-like tumors with high PD1 and PD-L1 expression [48].

It is generally believed that CD8+ T cells destroy tumor cells by binding to MHCI antigens [49], and the total number of CD8+ cells is positively correlated with tumor grade and better patient prognosis in BC [27]. Meanwhile, memory CD4+ T cells inhibit the outgrowth of tumor cells by promoting the proliferation of CD8+ cells [50]. The antitumor role of memory CD4+ T cells is also supported by previous evidence showing that increased disease-free survival of BC patients is directly related to an increase in activated memory CD4+ T cells [28]. Macrophages are an important type of immune cell in the tumor microenvironment and mainly include classically activated M1 macrophages and alternatively activated M2 macrophages [51]. Generally, the prooncogenic phenotype of M2-type macrophages promotes the occurrence and development of tumors by promoting tumor cell proliferation, inhibiting the tumor immune microenvironment, modulating matrix remodeling, and enhancing tumor angiogenesis [52–54]. In contrast, M1 macrophages are activated by Th1 cell factors; secrete inducible inductors, such as IL-12, iNOS, and TNF-*α*; and play a proinflammatory and antitumor role in the tumor microenvironment [29]. In our study, we demonstrated that the increased infiltrated immune cells in *RYR2*-mutant BC were all antitumorigenic immune cells, and CD8 T cells were positively correlated with activated memory CD4 T cells and M1 macrophages, while CD8 T cells, activated memory CD4 T cells, and M1 macrophages were negatively correlated with protumorigenic M2 macrophages. Thus, we suggest that the change in tumor-infiltrating immune cells induced by *RYR2* contributes to antitumor immunity in BC.

This research has some limitations. First, due to the lack of clinical data in the ICGC database, we could not determine whether *RYR2* mutations are also associated with prognosis and tumor immunity in European Union patients. Second, only informatics analyses were conducted in this study, and further experimental validations are needed. Third, we did not classify the different BC subtypes in this study. However, the mutated genes and immune infiltrating cells in different subtypes may be different [20, 55].

In summary, antitumor immune cells are suppressed in the tumor microenvironment, leading to a decrease in and low activity of antitumor immune cells among tumor-infiltrated cells [27, 56]. This is also the root cause of immunotherapy failure. In our study, we combined somatic gene mutation and TMB analyses and found that *RYR2* is frequently mutated in BC. *RYR2* mutation was related to higher TMB and better patient prognosis. More importantly, *RYR2* mutation induced an antitumor immune response. These findings reveal that *RYR2* mutation could serve as a biomarker to predict the immune response in BC.

## Figures and Tables

**Figure 1:** Overview of frequently mutated genes in BC. (a) Waterfall plot showing the top 30 mutated genes in TCGA BC cohort. Left panel: mutation frequency; right panel: different mutation types. (b) Waterfall plot showing the top 30 mutated genes in the ICGC BC cohort. Left panel: mutation frequency; right panel: different mutation types.

**Figure 2:** Gene mutations are correlated with TMB. (a) Venn diagram of the same frequently mutated genes in both TCGA and ICGC cohorts. (b) Mutated genes are correlated with a higher TMB. ^∗^*p* < 0.05; ^∗∗^*p* < 0.01; ^∗∗∗^*p* < 0.001; ns: no significance.

**Figure 3:** RYR2 mutation is associated with clinical prognosis. Kaplan-Meier curves of overall survival of the TMB-related mutated genes. The *p* value is marked in each plot.

**Figure 4:** Univariate (a) and multivariate (b) overall survival analyses of BC patients using a Cox proportional hazards model.

**Figure 5:** RYR2 mutation is associated with immune-related pathways. Gene enrichment plots showing that a series of immune-related pathways were enriched in the RYR2-mutant group. NES: normalized enrichment score. The *p* value is shown in each plot.

**Figure 6:** Distribution of tumor-infiltrating immune cells in BC samples. The stacked bar chart shows the distribution of 22 immune cells in each sample.

**Figure 7:** RYR2 mutation is associated with tumor-infiltrating immune cells. (a) Violin plot displaying the differentially infiltrated immune cells between the RYR2-mutant group and the RYR2-wild-type group. Blue represents the RYR2-wild-type group, and red represents the RYR2-mutant group. The *p* value is marked in the figure. (b) Correlation matrix of immune cell proportions. Red represents a positive correlation, and blue represents a negative correlation.

## Data Availability

The datasets generated and/or analyzed during the current study are available from the corresponding author on reasonable request. Data used included The Cancer Genome Atlas (TCGA, http://portal.gdc.cancer.gov/projects) and International Cancer Genome Consortium (ICGC, http://dcc.icgc.org/releases/current/Projects).

## Abbreviations

BC: Breast cancer
CTLs: Cytotoxic T lymphocytes
ER: Estrogen receptor
FDA: Food and Drug Administration
GSEA: Gene set enrichment analysis
HER2: Human epidermal growth factor receptor-2
ICGC: International Cancer Genome Consortium
RYR2: Ryanodine receptor 2
OS: Overall survival
PD-1: Programmed cell death receptor 1
PD-L1: Programmed cell death ligand 1
PR: Progesterone receptor
TCGA: The Cancer Genome Atlas
TMB: Tumor mutant burden
TNBC: Triple-negative breast cancer.

## Supplementary Materials

Supplementary Materials Supplementary File 1: detailed clinical information for this study.
